# Ferroptosis in Macrophage Impairment in Sepsis

**DOI:** 10.1155/2022/5792866

**Published:** 2022-09-20

**Authors:** Hongxuan Liu, Lei Li

**Affiliations:** Department of Emergency Internal Medicine, Shanxi Bethune Hospital, Shanxi Academy of Medical Sciences, Tongji Shanxi Hospital, Third Hospital of Shanxi Medical University, Taiyuan 030032, China

## Abstract

Sepsis is a clinical syndrome with high mortality, which can lead to multiple organ dysfunction syndrome. Nonspecific immune dysfunction and immune imbalance are its important pathological features. Macrophages are important immune cells and one of the important components of innate and adaptive immunity. Regulating the function of macrophages may be a potential method for the treatment of sepsis. Up to now, ferroptosis has been proved to be involved in the pathophysiological mechanism of many diseases, such as Alzheimer's disease, cancer, Parkinson's disease, and renal degeneration. At present, relevant studies have reported that ferroptosis may be involved in the occurrence of sepsis This paper reviews the existing mechanisms of iron ptosis in macrophages in sepsis, with a view to providing si'l for future studies on sepsis.

## 1. Introduction

Sepsis is one of the main causes of death in critically ill patients. Sepsis is a clinical syndrome with high mortality, which is caused by infection and leads to dysfunction of host response and life-threatening organ function damage [1]. A multicenter study shows that there are as many as 31million patients with sepsis worldwide every year, including 19.4 million cases of severe sepsis and about 6 million deaths [2]. The pathogenesis of sepsis is unknown. The change of immune function of the host after sepsis is an important reason affecting the prognosis. Whether in the process of innate immunity or adaptive immunity, macrophages play a crucial role in the infection of the body [3]. Ferroptosis is a new form of adaptive and programmed cell death first proposed by Brent r. Stockwell in 2012 [4]. Ferroptosis is a new type of programmed cell death that is iron dependent and different from apoptosis, cell necrosis, and autophagy. The main mechanism of iron death is that, under the action of divalent iron or ester oxygenase, it catalyzes the high expression of unsaturated fatty acids on the cell membrane to produce lipid peroxidation, thus inducing cell death. In addition, GPx4, the regulatory core enzyme of the antioxidant system, was also decreased. Ferroptosis is involved in the pathological process of a variety of diseases, including degenerative diseases, malignant tumors, stroke, and ischemia-reperfusion injury [5–7]. This article reviews the effect and mechanism of ferroptosis on the inflammatory effect of macrophages in sepsis.

## 2. Changes of Macrophages in Sepsis

Macrophages are an important part of immune cells in the body. They have the functions of secreting inflammatory cytokines, chemotaxis, phagocytosis, regulating inflammatory response, and killing microorganisms. When sepsis occurs, macrophages can be recognized by toll like receptors (TLR-4), thus, activate innate immunity. At the same time, t and B lymphocytes specifically recognize the antigen epitopes of T and B lymphocytes presented by antigen presenting cells (APCs) through cell receptors [8]. After recognizing the antigens, t and B lymphocytes, with the participation of costimulatory molecules, develop the effects of activation, proliferation, and differentiation [9]. Cells can be phagocytized and cleared by macrophages participating in adaptive immunity. Most of the macrophages in the tissues come from yolk sac or embryonic hematopoietic stem cells, which can change according to the change of microenvironment. Generally speaking, macrophages can be classified according to their function and activation, i.e., M1 (classical activation) or M2 (alternative activation), but the time point at which macrophages differentiate into M1 type macrophages and M2 type macrophages is not clear. M1 macrophages are mainly composed of lipopolysaccharide (LPS) and/or interferon *γ* (interferon *γ*), tumor necrosis factor *α* (tumor necrosis factor *α*), and other cytokines [10–12]. M2 macrophages are mainly composed of IL-4 and transforming growth factor *β* (transforming growth factor *β*) and immune complex induced activation [13]. M1 macrophages can release proinflammatory cytokines, inhibit cell proliferation around tissues, and cause tissue damage. M2 macrophages release anti-inflammatory cytokines, help cell proliferation, and promote wound healing and tissue repair [14]. M1 and M2 types of macrophages can be converted to each other under certain conditions, so that differentiated macrophages can “repolarize” and play corresponding functions [15]. Macrophages continuously monitor the body's immune defense, which requires continuous energy supply [16]. Under normal physiological conditions, macrophages take oxidative phosphorylation of glucose as their main metabolic pathway for energy demand. When sepsis occurs, the body's hypoxia attack leads to the disorder of glycolysis pathway [17]. The imbalance of macrophage polarization into M1 or M2 has an adverse impact on the body, and its metabolism changes in a stress manner, affecting the inflammatory response and the function of the immune system.

The expression of genes related to glycolysis in macrophages was enhanced during the excessive inflammatory response phase of sepsis, but decreased during the immune tolerance phase. Studies have shown that after LPS stimulated macrophages, rapamycin target protein, and hypoxia inducible factor-1*α* (hypoxia-inducible factor-1 *α*, HIF-1*α*). Increased expression can promote the expression of glycolysis-related genes and increase the expression of fructose-2-kinase 6-phosphate, thereby promoting aerobic glycolysis [18]. After LPS activated macrophages, the expression of inducible nitric oxide synthase increased, and the activity of some target proteins in mitochondrial electron transport chain. The activity decreases, thereby inhibiting the tricarboxylic acid cycle and oxidative phosphorylation [19]. After the metabolic changes of macrophages, their metabolic intermediates affect the function of immune cells. In the sepsis mouse model, it was found that by preventing HIF-1*α*, it may regulate the harmful immune metabolism in macrophages and become a new idea of immunotherapy for sepsis [20].

Autophagy is an important way for the body to remove harmful substances such as abnormal organelles, pathogens, misfolded, or aggregated proteins, and it is one of the main mechanisms to maintain the homeostasis of the intracellular environment. Studies have shown that autophagy can regulate the release of inflammatory cytokines, and autophagy reduction will promote inflammatory response and lead to cell death [21]. The enhancement of macrophage autophagy can play a protective role by negatively regulating the abnormal activation of macrophages, regulating the polarization typing of macrophages, reducing the activation of inflammatory bodies and the release of inflammatory cytokines, and affecting the apoptosis of macrophages. Its level determines the development and prognosis of sepsis to a certain extent.

In sepsis, the polarization of macrophages is closely related to metabolism and autophagy. Glucose metabolism provides energy for macrophage typing and autophagy to promote the elimination of pathogens. Autophagy level changes with the change of macrophage phenotype, reducing systemic inflammatory response. To further understand the functional changes and mechanisms of macrophages in sepsis, intervention on macrophage function may become a new method for the treatment of sepsis.

## 3. Effect of Ferroptosis on Anti-Inflammatory Activity of Macrophages

### 3.1. Regulation of Macrophage Inflammatory Cytokine Levels

Sepsis is characterized by extensive inflammation after host infection, resulting in a storm of cytokines. Excessive activation of inflammatory cytokines eventually leads to systemic inflammatory response syndrome (SIRS). The level of inflammatory cytokines affects the development and prognosis of sepsis to a certain extent. During sepsis, many proinflammatory IL-1 in cytokines *β*, IL-6, and TNF-*α* plays an important role in the prognosis of patients. IL-1*β* levels were reported to be higher in patients who died during sepsis than in survivors, and TNF-*α* was associated with the severity of the infection, suggesting to some extent that high levels of IL-1*β* and TNF-*α* were negatively associated with the prognosis of sepsis [22].

In vitro studies in mice have shown that ferroptosis can significantly reduce the proinflammatory cytokines secreted by macrophages induced by LPS, such as TNF-*α*, IL-6, and IL-8 [23]. Cao et al. [24] found that ferroptosis can significantly inhibit IL-1 after LPS induced mouse bone marrow-derived macrophages *β*, TNF-*α*, and IL-6, thereby alleviating systemic inflammatory response. Zhang et al. [25] confirmed that ferroptosis can reduce the inflammatory cytokine IL-1 in the mouse model *β* horizontal effect. Li et al. [26] showed that ferroptosis can reduce the risk of traumatic brain injury in mouse models IL-1 *β*, TNF-*α*, and IL-6. High mobility group B1 (HMGB1) is also a key proinflammatory cytokine. Its level in late sepsis is closely related to the mortality of sepsis patients. The inhibitory effect of ferroptosis on macrophage inflammatory cytokines may be partly due to its anti-inflammatory effect in sepsis. Studies have shown that the use of a single inflammatory cytokine antagonist does not improve the prognosis of patients with sepsis, but it may improve the prognosis of sepsis by interfering with the overall cytokine level. At present, it is believed that macrophages can reduce the mortality of patients and protect organs by inhibiting the expression of a variety of inflammatory cytokines.

### 3.2. Effect Macrophage Polarization

M1/M2 markers are closely related to the development and prognosis of sepsis. M1 macrophages play an important role in the early progression of sepsis. IFN-*γ* can inhibit the transformation of macrophages to M1 type. Juan et al. [27] showed IFN-*γ*. In the secretion experiment, ferroptosis could reduce IFN-*γ* protein expression level. Wang et al. [28] found that ferroptosis can reduce IFN-*γ* MRNA expression level. This study suggests that ferroptosis may reduce IFN-*γ*. The expression level affects the polarization of macrophages, thus playing the role of anti-inflammatory response. Li et al. [5] showed that ferroptosis passed *α* 2 adrenergic receptor signal mediates the increase of the transcription level of M2 markers arg1 and CD206. The above studies show that ferroptosis can reduce the release of inflammatory cytokines and multiple organ damage by inhibiting the polarization of M1 macrophages and promoting the polarization of M2 macrophages.

### 3.3. Effect Macrophage Metabolism

Cellular energy metabolism plays an important role in the function of immune cells in sepsis. It is of great significance to study its mechanism and regulation for revealing the pathophysiological mechanism of sepsis. HIF-1*α* is generally not expressed, but can be induced by LPS activated macrophages. When LPS stimulated macrophages, HIF-1*α* increased expression of genes related to glycolysis, so as to promote aerobic glycolysis and finally increase the expression of inflammatory cytokines (such as IL-1*β*, TNF, and HMGB-1), activate systemic inflammatory response, and cause multiple organ dysfunction [29]. Li et al. [30] found that HIF-1 in myeloid cells *α* deletion can significantly reduce TNF-*α* expression of succinic acid and glutamine, as important intermediates of glucose metabolism, and can improve glucose metabolism in sepsis. Studies have shown that succinic acid and glutamine can directly or indirectly increase HIF-1*α* level and stability and promote the production of inflammatory cytokines [31]. So far, the research on the effect of ferroptosis on succinic acid is not clear. Considering that both glutamine and succinic acid are related to HIF-1*α*. Therefore, it can be assumed that ferroptosis may inhibit HIF-1*α* [32]. It indirectly affects succinic acid and glutamine and provides energy for anti-inflammatory of macrophages. This hypothesis requires a large number of experimental studies to prove. It is worth paying attention to whether ferroptosis has a direct effect on succinic acid and glutamine.

### 3.4. Effect Macrophage Autophagy

Autophagy of macrophages is closely related to related key proteins, and signaling pathways, such as Jun signaling pathway, PI3K/AKT signaling pathway, and NF-*κ* B signaling pathway, play an important role in the activity of macrophage autophagy [29]. Wei et al. [33] and Wang et al. [34] showed that ferroptosis can reduce LPS induced acute lung injury and autophagy through PI3K/AKT/mTOR signaling pathway. Xie et al. [35] studied ferroptosis regulated autophagy related proteins and found that after LPS treatment, the expression levels of LC3 II and beclin-1 decreased and the expression of p62 increased. After ferroptosis intervention, the expression levels of LC3 II/LC3 and beclin-1 increased significantly and the expression of p62 decreased. Fang et al. [36] showed that ferroptosis could enhance autophagy by inhibiting PI3K, downregulate the expression of beclin-1, upregulate the expression of p62, and reduce the ratio of LC3 II/LC3 I, thus reducing the inflammatory response of macrophages induced by LPS. After neuronal apoptosis, ferroptosis treatment can significantly downregulate the mRNA and protein expression levels of beclin-1 and LC3 II/lc3 I, inhibit autophagy, and play an organ protective role [37]. Under normal circumstances, the autophagy level of the body is low. It will be stimulated under stress, inflammation, and hypoxia to enhance the body's defense function. However, excessive autophagy will cause autophagic death of macrophages and increase inflammatory reaction [38]. Beclin-1, LC3, and p62, as important marker proteins of macrophage autophagy, play an important role in the autophagy defense mechanism of the body [39]. The above studies show that ferroptosis can affect the expression levels of these three proteins induced by LPS, but whether it can enhance or inhibit autophagy has not been recognized and needs further study. The changes of macrophage autophagy level in different stages of sepsis are complex. There are still few studies on the key points of ferroptosis affecting autophagy and playing an anti-inflammatory role. If the right time is accurately selected and the autophagy level is regulated by ferroptosis, the mortality of sepsis may be effectively reduced.

## 4. Discussion

With the continuous development of medicine, sepsis, as one of the diseases with the highest mortality in the world, is still a difficult problem for clinicians to overcome because of its long treatment cycle and lack of specificity. The underlying pathogenesis of sepsis is not yet clear. It involves complex systemic inflammatory network effects, gene polymorphisms, immune dysfunction, abnormal coagulation function, tissue damage, and abnormal response of the host to different infectious pathogenic microorganisms and toxins. It is closely related to the pathophysiological changes of multiple systems and organs. The pathogenesis of sepsis still needs further elucidation.

Macrophages, as one of the important members involved in inflammatory response, play an irreplaceable role in sepsis. Influence of ferritinase on the inflammatory activity of macrophages. Exploring whether ferroptosis can affect other functions and mechanisms of macrophages, that is, further targeting the release of macrophage inflammatory cytokines, metabolic pathways, and the strength of autophagy and signal pathways, is of great significance to find more targets for the treatment of sepsis.

The most effective way to treat and prevent sepsis is to treat and prevent sepsis on the basis of its pathogenesis. Unfortunately, the pathogenesis of sepsis has not yet been fully clarified. In this case, we should do a good job in all aspects of clinical prevention according to the causes of sepsis and strive to reduce the risk factors of inducing infection, which plays an important role in the treatment and prevention of sepsis. With the progress of medical research, large sample and multicenter clinical randomized controlled study will bring more evidence-based medical evidence for the treatment of sepsis. The elucidation of sepsis mechanism in the future will certainly bring new hope for the treatment and prevention of sepsis.

## 5. Conclusion

In sepsis, macrophages undergo a series of changes. Moreover, the anti-inflammatory activity of macrophages caused by ferroptosis will also have a series of effects on the level of inflammatory cytokines, the polarization of macrophages, the metabolism of macrophages, and the autophagy of macrophages. This may suggest that the damage of macrophages in sepsis is related to ferroptosis, which provides a way of thinking for studying the mechanism of sepsis.

## Data Availability

The data used to support this study is available from the corresponding author upon request.
